The article "MHA-Net: A Multibranch Hybrid Attention Network for Medical Image Segmentation" was published in 2022. Journal: Comput Math Methods Med.

# MHA-Net: A Multibranch Hybrid Attention Network for Medical Image Segmentation

**DOI:** 10.1155/2022/8375981

**Published:** 2022-10-06

**Authors:** Meifang Zhang, Qi Sun, Fanggang Cai, Changcai Yang

**Affiliations:** ^1^Department of Health Management, Fujian Health College, Fuzhou 350101, China; ^2^College of Computer and Information Science, Fujian Agriculture and Forestry University, Fuzhou 350002, China; ^3^Department of Vascular Surgery, the First Affiliated Hospital, Fujian Medical University, Fuzhou 350005, China

## Abstract

The robust segmentation of organs from the medical image is the key technique in medical image analysis for disease diagnosis. U-Net is a robust structure for medical image segmentation. However, U-Net adopts consecutive downsampling encoders to capture multiscale features, resulting in the loss of contextual information and insufficient recovery of high-level semantic features. In this paper, we present a new multibranch hybrid attention network (MHA-Net) to capture more contextual information and high-level semantic features. The main idea of our proposed MHA-Net is to use the multibranch hybrid attention feature decoder to recover more high-level semantic features. The lightweight pyramid split attention (PSA) module is used to connect the encoder and decoder subnetwork to obtain a richer multiscale feature map. We compare the proposed MHA-Net to state-of-art approaches on the DRIVE dataset, the fluoroscopic roentgenographic stereophotogrammetric analysis X-ray dataset, and the polyp dataset. The experimental results on different modal images reveal that our proposed MHA-Net provides better segmentation results than other segmentation approaches.

## 1. Introduction

The robust organ segmentation from medical images is essential for medical image analysis. Its critical task is to segment objects of interest (e.g., lesions or organs) in medical images, providing important significance and value for accurate identification, rational diagnosis, prediction, prevention of diseases, etc. However, medical image segmentation is still a significantly tricky task because of the poor quality of medical images with a low signal-to-clutter ratio. In addition, organs of interest are often buried in complex backgrounds with muscles, blood vessels, bones, etc.

Many traditional medical image segmentation approaches have been proposed in the past decades. Massoptier and Casciaro [1] used the level set method to compute a smoother liver surface and then adopted automatic classification to detect the hepatic lesions. A semiautomatic level set method, which includes the spiral-scanning approach and the statistical pixel classification method, was proposed by Smeets et al. [2] for liver tumors combining segmentation. A multiconcavity modeling vessel segmentation method, which combines both line-shape concavity measure and locally normalized concavity measure, was proposed by Lam et al. [3]. Azzopardi et al. [4] proposed trainable COSFIRE filters for retinal vessel image segmentation. The common drawback of the traditional supervised learning image segmentation algorithms is that they depend on accurate and complex feature extraction. The modeling and selection of these features require not only professional knowledge but also difficulty to obtain, which makes the quality of the feature model directly impact image segmentation and classification, thus affecting the versatility and accuracy of the algorithm.

The article "MHA-Net: A Multibranch Hybrid Attention Network for Medical Image Segmentation" was published in 2022. Journal: Comput Math Methods Med.

With the development of machine learning in image and video analyses, feature automatic learning methods using convolutional neural networks (CNN) have become a viable method for medical image segmentation. Unlike classic pixel classification methods that typically utilize hand-crafted image features, CNN methods learn image features and solve hand-crafting problems. The U-Net [5] is one of the well-known medical image segmentation network structures, showing superior performance in neuronal structure segmentation and cellular segmentation. The U-Net that fuses feature maps from different stages by hopping connections is an encoder-decoder model. The spatial dimensionality of the feature maps is progressively reduced by using the encoder. Then, more high-level semantic features can be obtained. The decoder is used to find the details and spatial dimensions of the medical image. Wang et al. [6] built an efficient dual encoder U-Net (DEU-Net) to improve the pixel-to-pixel segmentation performance of retinal vessels. Alom et al. [7] developed a novel recurrent residual U-Net (R2U-Net), which has shown good performance in many biomedical image applications. Wu et al. [8] presented a Vessel-Net, which combines the perceptual and residual models for medical image segmentation. Yang et al. [9] proposed a retinal vessel segmentation model (MSFFU-Net) incorporating the multiscale features. Samuel and Veeramalai [10] proposed a two-stage vessel segmentation method to selectively learn the appropriate blood vessels. Xu et al. [11] developed a dual-context network for segmenting medical images aggregating multiscale and global contexts. In this network, the global context is recovered using the global context transformer consisting of a new adaptive context fusion module which is proposed to capture the global context. Lachinov et al. [12] proposed projective skip connections between an encoder and a decoder to address medical image segmentation problems in the subset of dimensions. These CNN-based approaches have achieved good performances. However, the consecutive downsampling encoders of FCN-based U-Net and its varieties result in the loss of contextual information and insufficient recovery of high-level semantic features during upsampling, which is not conducive to medical image segmentation. Khan et al. [13] developed a deep hybrid network (DH-Net), which combines DenseNet with U-Net, to classify the land cover in satellite images. DenseNet builds the multiple-scale feature extraction. Khan et al. [14] proposed an encoder-decoder network (EE-Net) to detect the building footprints in satellite images. These two methods have achieved good results in remote sensing image segmentation, but the effectiveness of medical image segmentation needs to be further verified.

The article "MHA-Net: A Multibranch Hybrid Attention Network for Medical Image Segmentation" was published in 2022. Journal: Comput Math Methods Med.

In this study, we explore a new multibranch hybrid attention network (MHA-Net) for medical image segmentation that can recover more high-level semantic features. The proposed MHA-Net mainly consists of an encoder module with the pretrained ResNet, a lightweight pyramid split attention (PSA) [15], and a novel multibranch hybrid attention (MHA) feature decoder module. The U-Net lacks the ability to integrate the multiscale context due to consecutive convolution and pooling operations in the decoders. We use PSA as a bridge to connect the encoder and decoder to recover more multiscale spatial information by infusing four groups with a multiscale pyramid convolution structure. The proposed MHA block could recover more high-level semantic information by adopting concatenation and summation operations with the corresponding feature maps. The contributions of this paper can be listed as follows.

Firstly, we propose a novel multibranch hybrid attention feature decoder to recover more high-level semantic features.

Secondly, we propose an MHA-Net for medical image segmentation, which contains a feature encoder, a lightweight PSA connecting the encoder and the decoder, and our proposed multibranch hybrid attention feature decoder.

Finally, the experimental results on the DRIVE dataset, the fluoroscopic roentgenographic stereophotogrammetric analysis (FRSA) X-ray dataset, and the polyp dataset compared with the standard segmentation methods show that our proposed MHA-Net is better.

## 2. MHA-Net

Figure 1 illustrates the schematic of the proposed MHA-Net. It contains a feature encoder block, a feature decoder block, and a multiscale PSA module that connects the encoder and decoder subnetworks. Next, we describe each part of the proposed MHA-Net in details.

### 2.1. Feature Encoder Block

The encoder block in U-Net consists of two 3 × 3 convolutions with a ReLU and a 2 × 2 max pooling. In this paper, following the Ce-Net [16], a pretrained ResNet-34 [17] is used as the feature encoder block. The pretrained weight parameters on the ImageNet dataset are used as parameter initialization.

The article "MHA-Net: A Multibranch Hybrid Attention Network for Medical Image Segmentation" was published in 2022. Journal: Comput Math Methods Med.

### 2.2. PSA

To obtain more multiscale spatial information and high-level semantic information from the medical image, the lightweight PSA module [15] is used as a bridge to connect the encoder and bottom of decoder subnetworks. The feature map of the encoder is split into four groups, and each group has 128 channels. Following [15], the convolution kernel parameters are set to be 3, 5, 7, and 8. And the group convolution parameters are set to be 1, 4, 8, and 16. A multiscale pyramid convolution structure, which can more accurately merge adjacent scales of context features, is adopted to integrate the feature of different-scale feature maps on each channel. The channel attention weight of the multiscale feature map is obtained by using the SEWeight module [18]. Then, the crossdimensional interactions can be established. The attention weights of the correlated channels, which establish the remote channel dependencies, are recalculated by using the Softmax operation. Finally, the multiscale feature maps are multiplied with the corrected attention vectors to extract a richer multiscale feature map passed to the feature decoder block.

### 2.3. Proposed Feature Decoder Block

In U-Net, the decoder block contains an upsampling operation, a concatenation operation, and two convolutions with a ReLU. The concatenation operation uses the skip connection to capture some context from the encoder. However, unlike the U-Net, the proposed decoder consists of our multibranch hybrid attention block, which can recover more high-level semantic features. A novel feature decoder, which contains a multibranch hybrid attention (MHA) block, a transposed convolution, and two 3 × 3 convolutions, is proposed. Our proposed MHA block contains a transposed convolution, a concatenation with the correspondingly cropped feature maps, two 3 × 3 convolutions, channel attention, and a summation with the corresponding cropped feature maps consecutively. The architecture of the multibranch hybrid feature decoder with an 800 × 800 × 3 input data size is shown in Figure 2. The 25 × 25 × 512 feature map is input into the proposed feature decoder. We use a transposed convolution to upsample the feature map and obtain a feature map with a 50 × 50 × 512 size. Then, this feature map and its corresponding feature map from the feature encoder are concatenated and a feature map with a 50 × 50 × 768 size can be obtained. Two 3 × 3 convolutions and channel attention are used to selectively weigh each channel's significance, and a feature map with a 50 × 50 × 256 size is obtained. After that, we make a summation operation between it and its corresponding feature map from the feature encoder. We obtain a feature map with a 100 × 100 × 384 size. After the other three multibranch hybrid attention blocks, we obtain a feature map with a 800 × 800 × 32 size. Finally, the segmentation result is obtained using two 3 × 3 convolution operations.

The article "MHA-Net: A Multibranch Hybrid Attention Network for Medical Image Segmentation" was published in 2022. Journal: Comput Math Methods Med.

## 3. Experimental and Discussion

To verify the proposed MHA-Net performance for medical image segmentation, we test it on the DRIVE dataset [19] and the FRSA X-ray dataset [20]. The DRIVE dataset contains 20 trained and 20 tested retinal images with a 584 × 565 × 3 size. The FRSA X-ray dataset includes 76 trained and 26 tested images with a 800 × 800 × 3 size. To evaluate the generalization ability of the proposed MHA-Net, we adopt the polyp dataset, which contains Kvasir [21], ClinicDB [22], and ColonDB [23] datasets. The Kvasir, ClinicDB, and ColonDB datasets contain 1000, 612, and 380 images, respectively. Following [24], we use 90% of Kvasir and ClinicDB data as a training set, the remaining 10% as a validation set, and the ColonDB dataset as a test set. The size of all polyp data is set to 352 × 352 × 3. In this paper, we use the binary crossentropy as the loss function. We use the batch size of 4 for the DRIVE dataset, 4 for the FRSA X-ray dataset, and 8 for the polyp dataset. We adopt the Adam optimizer with initial learning rate 0.0001 to optimize all models. We set the epoch to 300 for the DRIVE dataset and 150 for the FRSA X-ray dataset and polyp dataset. The parameter size of the proposed MHA-Net is 34.79 M.

### 3.1. Experimental with DRIVE Data

The proposed MHA-Net is compared to U-Net [5], JSPL-Net [25], Ce-Net [16], IterNet [26], AGAC-Net [27], DAP [28], and VSSC-Net [10]. In this paper, three common performance measures, area under the receiver operating characteristic curve (AUC), sensitivity (Se), and accuracy (Ac), are adopted as standards for our evaluation in retinal image segmentation.

Table 1 presents the values of the quality of AUC, Se, and Ac for each medical image segmentation method. Table 1 shows that our proposed MHA-Net provides the best segmentation performances in light of AUC, Se, and Ac. For example, the AUC score of our proposed MHA-Net is 0.9864 and is over 0.9834, 0.9752, 0.9831, 0.9813, 0.9847, 0.9788, and 0.9789, given by the U-Net, R2U-Net, Ce-Net, Ce-Net, IterNet, AGAC-Net, DAP, and VSSC-Net methods. We can find similar results for Se and Ac scores.

Figure 2 shows segmentation results by different approaches on DRIVE images. Column 1 in Figure 2 shows two original retinal images. Columns 2–4 in Figure 2 show the corresponding segmentation results provided by U-Net, Ce-Net, and our proposed MHA-Net, respectively. Column 5 in Figure 2 show the ground truth. Carefully observing Figure 2, we can find that the segmentation results given by our proposed MHA-Net are superior to that provided by U-Net and Ce-Net. For example, our proposed MHA-Net provides a little better segmentation accuracy, as shown in the red circled region in Figure 2.

The article "MHA-Net: A Multibranch Hybrid Attention Network for Medical Image Segmentation" was published in 2022. Journal: Comput Math Methods Med.

### 3.2. Experimental with FRSA X-Ray Data

The proposed MHA-Net is compared to U-Net [5], Ce-Net [16], RSAN [29], and SA-UNet [30]. In this section, three common performance measures, Dice coefficient (DC), intersection ratio (IR), and Ac, are used as standards for our evaluation of X-ray image segmentation:

(1) $$\begin{array}{c} \text{DC}=\frac{2\times \text{TP}}{\left(\text{TP}+\text{FP}\right)+\left(\text{TP}+\text{FN}\right)},\\ \text{IR}=\frac{\text{TP}}{\text{TP}+\text{FN}+\text{FP}}. \end{array}$$

Table 2 gives the values of the quality of DC, IR, and Ac on the FRSA X-ray images for different segmentation methods. Table 2 shows that our proposed MHA-Net provided the best segmentation performances in terms of DC, IR, and Ac scores. The DC score of our proposed MHA-Net is 0.9645 and is over 0.9264, 0.9623, 0.9389, and 0.9204, respectively, obtained by the U-Net, Ce-Net, RSAN, and SA-UNet methods. We can find similar results for IR and Ac scores.

Column 1 in Figure 3 shows two original stent images. Columns 2–6 of Figure 2 show the stent segmentation results by U-Net, Ce-Net, RSAN, our proposed MHA-Net, and the ground truth. The segmentation effect of our MHA-Net is better than that given by U-Net, Ce-Net, and RSAN. For example, our proposed MHA-Net provides a little better segmentation accuracy, as shown in the red-circled region in Figure 3.

### 3.3. Experimental with the Crossdataset

The proposed MHA-Net is compared to U-Net [5], UNet++ [31] Ce-Net [16], PraNet [24], and HarDNet-MSEG [32]. In this section, eight common performance measures, Recall(Rec), Specificity(Spec), Precision(Prec), DC, IoU_poly(IoUp), IoU_bg(IoUb), IoU_mean(mIoU), and Ac, are used as standards for our evaluation in polyp image segmentation:

(2) $$\begin{array}{c} \text{Rec}=\frac{TP}{\text{TP}+\text{FN}},\\ \text{Spec}=\frac{\text{TN}}{\text{TN}+\text{FP}},\\ \text{Prec}=\frac{\text{TP}}{\text{TP}+\text{FP}},\\ \text{IoUp}=\frac{\text{IoUp}}{\text{TP}+\text{FP}+\text{FN}},\\ \text{IoUb}=\frac{\text{TN}}{\text{TN}+\text{FP}+\text{FN}},\\ \text{mIoU}=\frac{\text{IoUp}+\text{IoUb}}{2.0}. \end{array}$$

We verify the model's generalization ability on Kvasir [21], ClinicDB [22], and ColonDB [23].  Table 3 presents the values of quality of Rec, Spec, Prec, DC, IoUp, IoUb, mIoU, and Ac on the polyp images for different segmentation methods.  Table 3 shows that the proposed MHA-Net provided the best segmentation performances in terms of scores of Rec, DC, IoUp, IoUb, mIoU, and Ac. For Spec and Prec metrics, HarDNet-MSEG achieves the best results, followed closely by U-Net and the proposed MHA-Net.  Table 3 shows that the proposed MHA-Net has good model generalization ability.

The article "MHA-Net: A Multibranch Hybrid Attention Network for Medical Image Segmentation" was published in 2022. Journal: Comput Math Methods Med.

### 3.4. Ablation Study

To evaluate the effectiveness of individual components in the proposed MHA-Net, we performed ablation experiments on the femoral-popliteal stent dataset. We refer to the network without PSA, channel attention (SE), and summation (Sum) operation as our baseline.  Table 4 shows that comparing the baseline with the PSA module can improve the DC, IR, and Ac indicators, showing that the proposed PSA module captures rich multiscale features. Combining the channel attention to compare the baseline can also improve the DC, IR, and Ac metrics. Channel attention values useful features while suppressing ones not important to the current task. Combining the PSA module, the SE module, and the Sum operation, our network can obtain the best performance and Sum operation can obtain more advanced semantic information.

### 3.5. Failure Cases

The proposed MHA-Net does not successfully address all cases of medical segmentation problems.  Figure 4 shows the segmentation results of the ColonDB dataset. The proposed MHA-Net does not segment polyps very well, as shown in Figure 4. In polyp data, the size and shape of the lesion vary greatly. Moreover, the boundary of the lesion area is often blurred due to the low contrast between the lesion area and the surrounding area. This problem is not well addressed using our proposed model. However, this issue also affects most other state-of-the-art image segmentation methods.

## 4. Conclusions

In this study, we propose the multibranch hybrid attention feature decoder block and present an MHA-Net for medical image segmentation. Experimental results on DRIVE dataset, FRSA X-ray dataset, and polyp dataset show that our MHA-Net is superior to other segmentation approaches, including U-Net [5], JSPL-Net [25], Ce-Net [16], IterNet [26], AGAC-Net [27], DAP [28], VSSC Net [10], UNet++ [31], PraNet [24], and HarDNet-MSEG [32]. The multibranch hybrid attention feature decoder of the proposed MHA-Net can recover more high-level semantic features.

## Figures and Tables

**Figure 1:** The proposed MHA-Net with a 800 × 800 × 3 input data size. The proposed MHA-Net contains a feature encoder block, the proposed MHA decoder block, and a PSA module that connects the encoder and decoder subnetworks.

The article "MHA-Net: A Multibranch Hybrid Attention Network for Medical Image Segmentation" was published in 2022. Journal: Comput Math Methods Med.

**Figure 2:** Retinal images and segmentation results provided by different approaches.

**Figure 3:** FRSA X-ray images and segmentation results provided by different approaches.

**Figure 4:** Examples show that our model cannot fully segment medical images.

**Table 1:** AUC, Se, and Ac Values on the DRIVE dataset by difference methods.

Method	Year	AUC	Se	Ac
U-Net [5]	2015	0.9834	0.8059	0.9627
JSPL-Net [25]	2018	0.9752	0.7653	0.9542
Ce-Net [16]	2019	0.9831	0.8330	0.9542
IterNet [26]	2020	0.9813	0.7791	0.9574
AGAC-Net [27]	2020	0.9847	0.7941	0.9558
DAP [28]	2021	0.9788	0.8227	0.9545
VSSC-Net [10]	2021	0.9789	0.7827	0.9627
Our approach	2022	*0.9864*	*0.8412*	*0.9636*

**Table 2:** DC, IR, and Ac values of difference segmentation methods on the FRSA X-ray dataset.

Method	Year	DC	IR	Ac
U-Net [5]	2015	0.9264	0.8678	0.9980
Ce-Net [16]	2019	0.9623	0.9276	0.9990
RSAN [29]	2020	0.9389	0.8848	0.9985
SA-UNet [30]	2021	0.9204	0.8525	0.9980
Our approach	2022	*0.9645*	*0.9325*	*0.9992*

**Table 3:** Eight standard performance measure values of different segmentation methods on the polyp dataset.

Method	Rec	Spec	Prec	DC	IoUp	IoUb	mIoU	Ac
U-Net [5]	0.6530	0.9940	0.8760	0.6481	0.5762	0.9564	0.7663	0.9588
UNet++ [31]	0.7705	0.9565	0.6375	0.6385	0.5401	0.9460	0.7431	0.9481
Ce-Net [16]	0.8129	0.9701	0.8167	0.7569	0.6873	0.9471	0.8172	0.9504
PraNet [24]	0.7820	0.9862	0.8110	0.7435	0.6644	0.9607	0.8126	0.9635
HarDNet-MSEG [32]	0.5886	*0.9988*	*0.9255*	0.6490	0.5736	0.9563	0.7649	0.9578
Our approach	*0.8000*	0.9905	0.8618	*0.7692*	*0.6982*	*0.9640*	*0.8311*	*0.9656*

**Table 4:** Ablation experiments on the femoropopliteal stent dataset.

Baseline	PSA	SE	Sum	DC	IR	Ac
✓				0.9581	0.9203	0.9990
✓	✓			0.9624	0.9282	0.9991
✓		✓		0.9614	0.9262	0.9991
✓	✓	✓	✓	0.9645	0.9325	0.9992

## Data Availability

The segmentation results for the proposed method data used to support the findings of this study are included in the article.
